# New Challenges for Ethics: The Social Impact of Posthumanism, Robots, and Artificial Intelligence

**DOI:** 10.1155/2021/5593467

**Published:** 2021-06-07

**Authors:** Lourdes Velázquez G

**Affiliations:** Centro Interdisciplinario de Bioética de la Universidad Panamericana (CIBUP), School of Medicine, Universidad Panamericana, Mexico City, Mexico

## Abstract

The ethical approach to science and technology is based on their use and application in extremely diverse fields. Less prominence has been given to the theme of the profound changes in our conception of human nature produced by the most recent developments in artificial intelligence and robotics due to their capacity to simulate an increasing number of human activities traditionally attributed to man as manifestations of the higher spiritual dimension inherent in his nature. Hence, a kind of contrast between nature and artificiality has ensued in which conformity with nature is presented as a criterion of morality and the artificial is legitimized only as an aid to nature. On the contrary, this essay maintains that artificiality is precisely the specific expression of human nature which has, in fact, made a powerful contribution to the progress of man. However, science and technology do not offer criteria to guide the practical and conceptual use of their own contents simply because they do not contain the conceptual space for the ought-to-be. Therefore, this paper offers a critical analysis of the conceptual models and the most typical products of technoscience as well as a discerning evaluation of the contemporary cultural trend of transhumanism. The position defended here consists of full appreciation of technoscience integrated into a broader framework of specifically human values.

## 1. Introduction

The current pandemic has represented a shocking and profound experience for humanity since it has brought to light conceptions concerning man, the world, and history that we can qualify as metaphysical but are not actually the result of philosophical reflections but rather structures of what Jung called the *collective unconscious* [1]. The role played by science and technology stands out as one of the most fundamental characteristics of this unconscious. We do not believe to be exaggerating by affirming that *technoscience* (as the close intertwining of science and technology is called nowadays) has achieved the place of supreme authority that guides us and almost imposes upon our way of life in our societies and the course of history.

In this paper, we will deal with this issue by considering the production of particularly significant *machines* from our point of view, i.e., those that in a broad sense fall within the field of *artificial intelligence* and *robotics*, as specific effects of technoscience, and we will reflect on the impact they have on the world of man.

This impact has long been considered essentially from an *ethical* point of view, i.e., by considering the *consequences* that the *use* of technoscience has had or can have on the human world and evaluating these consequences from a moral point of view. This is undoubtedly a matter of great importance, which concerns the very complex problem of the relationship between science and ethics and the reconciliation between freedom and responsibility of science. Therefore, we will devote some attention to this debate, which has produced the formation of two opposite fronts: *scientism* (which defends the unconditional value of technoscience and its growth) and *antiscience* (which rejects the value of science considering it a powerful dehumanizing factor). The position that we maintain is an intermediate path between these extremes and entails an analysis of the *artificial* as a domain, not opposite to the *natural*, but as an expression of the *specific nature* of man.

The next step will consist in examining a deeper theme, i.e., the one that ascribes technology with the aim of *improving* the nature of man himself by directly intervening on his nature. On closer inspection, it reveals an unconscious subversion of a thousand-year-old concept according to which man occupies an *intermediate* position between a lower level (where material bodies and animals belong) and a higher level (which is that of *spirituality* and the sacred). However, according to the new perspective, man continues to occupy an intermediate level but the highest one is made up of *machines.* Therefore, the *enhancement* of man and his world is placed in the growing measure in which he incorporates machines into the world which he lives in and even within himself. These are the theses which, to a more or less conscious extent, are characteristic of those contemporary cultural movements which are known by the names of *posthumanism* and *transhumanism*. The final part of this work will be dedicated to the discussion of these positions.

The relationship of the above considerations with the current COVID-19 pandemic is perhaps not immediately clear. Nevertheless, it is sufficient to consider how the general opinion, especially that diffused by the mass media, has indicated the availability of vaccines as the only decisive tool for “defeating” the pandemic, hailing the speed of vaccine production as a *miracle* of science. In the absence of this miracle (and its effective availability on a large scale), the only truly effective remedy enforced was the *isolation* of individuals with all its disastrous psychological, social, and economic consequences that we all know about. As well as having led to collective riots, isolation intolerability has fuelled the spread of antiscientific attitudes, conspiracy theories about the selfish interests of those who produce and recommend vaccinations, and even to the denial of the actual existence of the pandemic itself, and so on. All this has not only made it clear that human *vulnerability* is far from being limited to our physical health but also shows how it involves a very broad and articulated display of dimensions and values. For instance, we have already witnessed the emergence of solidarity stemming from the awareness that no individual survives alone and even less in a technologically advanced world. However, this is only the beginning of a profound reflection which, in particular, must dispel the childish illusion that once the virus will be defeated, we could *go back* to living as before. The authentic hope is that once this experience will be overcome, we will continue to live *better than before*, i.e., inspired by values capable of giving sense to our existence and which cannot be replaced by a process of increasing assimilation of men to machines.

## 2. The Ethical Dimensions of Science and Technology

A widespread tenet is that science must be *value-free*. This claim, eloquently expressed by Max Weber in the context of the social sciences, was intended to protect the *objectivity* of these sciences from the risk of becoming contaminated by the intrusion of the personal moral and social or political *values* of the investigator [2]. These values were believed to be strictly subjective and correspond to personal *options* of the scientist who, for this reason, had to abstain not only from expressing *value judgments* in the course of his *scientific* investigation but also from taking advantage of the results of the investigation in order to support his value options. This does not mean that science does not respect any values but that the values science is entitled (and obliged) to respect are only *cognitive values*, entailed by its being a search for *truth* by means of methodological criteria that can be summarized in the requirement of *objectivity.*

The same principles were later applied also to the natural sciences and found their expression in the thesis of the *neutrality of science*, widely debated last century, especially in the fifties and sixties. In the context of this debate, several scholars maintained that science must be objective and, therefore, free of any influence from “external” values, while other scholars upheld that science cannot and indeed must not remain neutral regarding such values. The debate was long and rather sterile since the discussants failed to distinguish two different aspects of science. On one hand, science is a system of *knowledge* whereas on the other hand, it is a complex system of *human activities*. It should be clear that from the first point of view, only cognitive values have the right to determine the acceptance or rejection of scientific statements or theories, while from the second point of view, scientific activity cannot dispense from responding to moral, social, political, economic, ecologic, and religious concerns that make up the *global sense* of any human activity on the personal and collective grounds.

The importance of this “external” dimension of science was made evident by several negative consequences of the development of *technology* and applied science that have shown that the *consequences* of technoscientific progress are by no means only beneficial to mankind but can entail disasters and serious risks for the survival of the present and also future generations. In other words, although technology must be guided by certain “internal” criteria of evaluation that can be summarized under the notion of *efficaciousness*, these criteria are not sufficient for a *global* evaluation not only of technology as a whole but also of single technological enterprises. Technology offers the most *efficient tools* for realizing pre-assigned *ends* but does not care and is not competent regarding the ethical *legitimacy* of the ends and even of the means proposed for the most efficient realization of the ends. Then again, precisely, these specific aspects are of great relevance for any *human activity*, so that humans are always confronted with the dilemma of whether *what can be done also ought to be done or not*. In this sense, ethics is inextricably included in the web of science and technology. This does not imply that we must stop scientific and technological progress but that it must be attuned to satisfy a wide spectrum of human values which can be attained if we adopt a *system-theoretic* approach where the technoscientific subsystem interacts with other social subsystems, each of which are defined by the pursuit of a legitimate goal. The mutual interdependence of these systems imposes *responsibility* on all social agents, including the scientific community, but at the same time, science is required to preserve its autonomy and be respected in its freedom of research since it pursues a genuine *value* that is essential for the general progress and flourishing of mankind. These precisions are useful in order to envisage a correct appreciation of the nature of the scope of the *artificial*.

## 3. The General Question of the Ethical Evaluation of Artificiality

In the context of ordinary discourse, the notion of “artificial” carries a negative connotation, as if what is artificial were in itself “not genuine.” In fact, it is often said that a certain attitude is “artificial” in the sense of not being spontaneous or sincere, and sometimes, “artificial” food is belittled with respect to “natural” food. At the base of this type of judgment is an implicit valuation of nature considered as intrinsically positive, genuine, and *good* in a very broad sense that is particularly reflected in the moral sphere. This opposition has deep ancient roots in Western culture since in ancient Greek, *art* (i.e., the product of human activities generally called *téchne*) was thought inferior to *nature* (the *phýsis*), considering art as an “imitation” of nature.

However, in the doctrine of the Stoics, nature becomes an absolute criterion of conduct and the maxim *sequere naturam* (follow your nature) appears as the supreme principle of moral life. This occurs because the natural *order*, which has always fascinated thinkers (regular succession of the seasons, of celestial phenomena, and of the life cycle of living beings), has shown itself as a rule that is reasonable and profitable to follow in order to achieve success in the most different forms of life and human activities. By extension, this very submission is considered optimum for living well within the *order* of society that was also perceived as a natural fact. Being born into this order of things, which preexists his entry into existence, each human being felt and thought of himself as part of Nature that surrounds him, includes him, and surpasses him. Therefore, people were led to believe that their dependence on nature was a fundamental condition of their own security and success in life. The Stoics added what we can call a religious meaning to this almost spontaneous perspective since they interpreted the natural order as the expression of the divine essence of the world and the consequence of the fact that the wisdom of an immanent Logos that determines the course of not only natural events but also human events that is realized in Nature.

When Christianity spread throughout the ancient world, it was inevitable that it absorbed the most influential conceptual elements of the Greek philosophical tradition of the time, especially certain aspects of Neoplatonic and Stoic thoughts. Consequently, it was spontaneous to interpret the Stoic vision according to a pattern of transcendence and consider the natural order as a reflection of divine will: at the top of this order stands God whose will and whose laws are expressed in the order of nature and society. Thus, it is easy to understand that ancestral man imposed (at the level of his intuition and instinctive ethos) the notion of authority and respect for the established order (whether of nature or of society) and that obedience was considered a fundamental virtue. The “Christianization” of this ancient perspective assured it a very long historical duration that lasted until the time of Western “secularization”, which took place in modern times.

Before going on to consider this transition, it is worth mentioning another more specifically philosophical reason that strongly contributed to the conception of moral precepts rooted in the respect for nature, i.e., the issue of finding a *rational justification* for moral norms that could guarantee their universality. Each moral norm can be synthesized in a “you must” and a reasonable being poses the question: “Why should I?” The answer cannot consist in indicating an authority or a constraint but rather a “reason” that, for example, would affirm that this duty corresponds to what defines the “goal” of man, but it can always be asked how we know that this is man's goal, and the final answer that many philosophers considered adequate is that the said purpose is *inscribed in the nature of man* and, therefore, does not depend on our choice or preference because it is something objective, universal, and immutable.

It should be noted that this type of reasoning dispenses with any religious reference, and in fact, in the 17th and 18th centuries, *natural law* and *natural ethics* (and even *natural religion*) theorists elaborated their doctrines without presupposing the acceptance of any religious faith. However, everyone knows that the adoption of respect for nature as the foundation of moral obligations has remained one of the most characteristic positions of the Catholic Church to date, although there are many theologians and moralists who have questioned the conformity of the Stoic perspective (i.e., the God-Nature-Man hierarchy) with the spirit of the biblical vision of a “Living God” who created man in His image and entrusted him with the task of submitting nature yet revealed Himself not in nature but in history. Then follows the evangelical vision of human life inspired by a hope which is dynamically oriented towards the future and committed to transforming the world under the impulse of the Spirit.

Precisely because this foundation of morality in nature continues to be defended by many authors, it is important to note, in view of the problem that interests us in this paper, that it is possible to admit that respect for nature represents a principle of morality without thereby rejecting the artificial. In fact, nature does not only include the “material” world but also the *human world*, and it is a specific characteristic of man that instead of guaranteeing his survival and development by “adapting himself to the environment” (as other living species do), he achieves this result “by adapting the natural environment to himself” and to his demands and needs, or rather, by building *an artificial world* that actually turns out to be his own *environment* or natural ecosystem, i.e., corresponding to his *specific human nature*. Consequently, the artificial as such cannot be morally condemned in the name of respect for nature, although it can be subjected to evaluation and moral limitation based on other ethical criteria. On the other hand, the idea that nature is always and unconditionally good for man is far from obvious, and man has always been forced to fight *against* exposure to nature as an “enemy,” no less than he has enjoyed the manifestations of friendly nature. Both these aspects represent the root of *technique*, which is the instrument that man, being endowed with reason and free will, has used to adapt the natural world to his demands, enjoying its friendly aspects and fighting against its hostile aspects.

The “traditional” picture has changed profoundly in the modern age, distinguished by the emergence of science in the modern sense and the ever-increasing value attributed to human freedom. The first characteristic has determined the transition from simple technique to *technology*, which can be considered as the branch of technique that consists in the application of scientific knowledge and allows an enormous development of the artificial in the creation of something truly new that stands next to the natural and *replaces* it many times.

So far, many issues have been raised and will be considered later on, but now, we are content to mention a few consequences of the scientific approach to nature. Nature is perceived as something that can and should be *manipulated* in order to *understand* it more deeply and also to be able to *enjoy* it: the “sacred” character that tradition attributed to it has been lost. Furthermore, scientific research shows us that material nature itself is not fixed and immutable since the earth, biological forms of life, and the universe itself have undergone historical development, as well as forms of social life, cultures, and human customs. This change in the common perception of the material world makes it very difficult to refer to nature as endowed with an intrinsic and immutable order. Nowadays, it appears to us much more similar to a display of complex interactions of a multitude of forces and structures that are the result of contingent history.

In this new vision, modernity places the accent on human freedom, which is no longer simply freedom of choice (or free will), but freedom of action that concerns the individual making himself a top priority. Firstly, modernity has emphasized this contemporary freedom and raised the problem of making it compatible with social limitations in a situation in which the very notion of natural social order is in crisis, and the concept of authority is rapidly deteriorating. Thus, men understand that just as they could intervene in the order of nature, they can intervene in the social order and even radically change it through revolutions without recognizing any sacred authority with a right to demand unconditional obedience and respect. In addition, man begins to feel authorized to intervene freely in the realities “built” by man himself (such as social institutions), but the development of human sciences (medicine, psychology, etc.) also allows the intervention on man himself and in a much more profound way than in the past. At this point, the problem of respect for nature reappears, and many are wondering whether freedom of intervention and modification can indeed be applied with respect to human nature (and today, they are also considering the limits that technological manipulation should reach in the case of nonhuman nature itself).

The considerations that we have presented force us to recognize that the moral positions still insisting on respect for nature are far from being a pure retrograde inheritance from a historically dead past since they contain a kernel of truth that cannot be ignored, although an absolutization of nature and its alleged immutability no longer appears defensible. The new accent on freedom of action is something that should be valued but without making it absolute, since the effort of all modern philosophical reflection in the ethical field has been to make the defence of this new freedom compatible with certain limitations that cannot be rejected.

## 4. A Space for Critical Reflection

After the arguments on the artificial and technoscience that we offered in the previous section, insisting that it makes no sense to contrast the artificial with the natural (since it is inscribed in the natural as well as being specific to human nature), it is necessary to underline that such an inscription is not automatic but requires *wise management* of the artificial so that it does not turn into a real threat to human nature itself. In other words, it is essential to open up a space for critical reflection on artificiality.

Therefore, excluding a priori the rejection of scientific research and technology in and of itself, there is rather an urgent need to reflect on the *goal* (for now still blurred) towards which the *utopia* of unlimited technological progress is driving us. Where will the paradisiacal path of technology lead to? Certainly, towards scenarios that have not yet been seriously discussed despite the work done by that philosophers, scientists, and even filmmakers who have foreshadowed them in an extraordinary way by issuing a cry of alarm that has remained unheard. We must be aware that the enthusiasm and uncritical identification of progress with technology obscures the hidden side of this kind of research, which, as in the field of automation, is even promising answers to the search for eternal life.

It has become a movement of public opinion that is captivating more and more people and scientists thanks to its subversive language and titanic vision in which the progress of technology is shown to be capable of upsetting society and transfiguring the human condition. There follows the risk of creating a dystopian society, divided into castes, in which only the super-rich will have the access to specific medical treatments aimed at physical enhancement, while the masses will be hypercontrolled, hyperconnected, and enslaved by a technocratic elite, thanks to the process of addiction described in the Overton window model. (The phenomenon of the variability of the attention and appreciation reserved for concepts and doctrines in different fields has been systematized in an interesting model known as the Overton window (after the name of its inventor, the sociologist Joseph Overton). Originally, proposed for the sociological analysis of politics, it is fruitfully applied in other fields as well: it presents six “windows” arranged according to an increasing order of degrees of acceptance, within which for example, a concept or opinion is found: unthinkable, radical, acceptable, sensible, popular, and policy. It can thus happen that a term, initially unknown and generally considered incomprehensible, begins to arouse curiosity, to enter speeches, to be taken seriously, and to become a fashionable label, even arousing a theorization, to the point of reaching a full legitimacy within a given disciplinary context. But the opposite can also happen, namely that a particularly authoritative and recognized term or doctrine in a certain discipline gradually descends the levels of Overton's windows. In virtue of this mechanism, even wrong and dangerous ideas can gradually and almost unconsciously become generally accepted, as it has pointed out, for instance in [3]. The model of Overton's window also finds application in the field of philosophy, and it would be easy to state examples.)

Faced with these issues, questions that are as simple as they are radical arise: are we sure that everything that is technologically possible (or that will be in the future) has to be researched and applied at all costs?

Today, research that until a few years ago would have been considered as despotic nightmares lies behind the word “progress” and is presented for public opinion as a goal for collective evolution. And if you dare criticize whatever is labelled as progress or advanced technology, you are automatically labelled and criticized as obscurantists and neo-Luddites, inhibiting confrontation and censoring dialogue.

Our purpose, therefore, is not to criticize *mechanization* or technological advancement which have improved living conditions and given relief to workers assigned to the most exhausting and dangerous tasks. If anything, our concern focuses on the ambiguous or even dangerous implications of these processes, from the risk of “deforestation of humans” to the degeneration of the “digital revolution.” Currently, man seems to have embarked on a new path towards a goal which was unimaginable only a few years ago: to become a *machine*. In fact, there are supporters of artificial intelligence who predict a future in which men and machines will merge into cyborgs: a real anthropological change, not only culturally but also in the understanding of man, nature, life, and the world [4].

At this point, we remember that not all *change is progress*, so it is legitimate to ask what can happen when the technological challenge goes beyond the unthinkable: when it launches into the senseless race for useless *high-tech* upgrades. The very paradigms of pro-life associations are at stake with the attempt to create a “perfect,” peaceful and technological society where there is no room for violence, uncontrolled emotions, or autonomous thinking and is inhabited by aseptic citizens of androgynous appearance. Moreover, their psychophysical balance is guaranteed by synthetic implants, and relationships are increasingly virtual producing increasingly lonely and depersonalized individuals.

## 5. Analyzing Some Facts

### 5.1. Technostress

It is true that computer technology unites us on the web, but very often, it can disconnect us from everyday life, also creating traps in a world where the *virtual reality* offered by computers, video games, social networks seems truer than *concrete reality*. Unfortunately, the side effects of this collective drive for progress have not yet been well-explored risking the creation of masses of technological idiots. Neuroscience has now proven that the human brain changes as a result of our interaction with the environment, and the less it exercises action, curiosity, memory, and critical spirit, the more it indulges in a sense of passive trust in the use of such electronic devices. In fact, the number of people obsessed with the constant control of smartphones is increasing, and we must, therefore, think about the harmful effects that the use of the Internet and smartphones has on behaviour and on the psyche. By virtue of the plasticity of our nervous system, the repetition of mental activities such as writing SMSs, chat messages, or checking emails strengthens some circuits in our brain, transforming those activities into rigid behaviours that are introjected as *habits* that can lead to pathologies, especially in younger people.

In fact, there is a disorder known as *technostress*, coined in 1984 by Craig Brod, linked to the massive and stratified use of new technologies. Technostress has been recognized in Italy as an occupational disease from the judge Raffaele Guariniello who was the first to impose this sentence in 2007 [5], which arises from the excessive and simultaneous use of digital information conveyed by video screens.

### 5.2. Isolation in the Virtual World

We, as adults, should also reflect on our responsibilities: the technological abuse that the new generations are suffering from is a form of compensation due to the lack of attention that we adults should have given them. It is a surrogate that can be addictive and cause permanent damage. One of the most disturbing phenomena, for example, is what in Japanese is called “Hikikomori boys” (i.e., “boys who stay secluded”). It consists of locking themselves in their room where they spend time on the Internet or play video games, basically running away from the real world to take refuge in the virtual one. The Hikikomori, aged between 12 and 30, do not leave home, are unable to manage their emotions, and end up living isolated in their bedrooms for months or years. As a result, they begin to feel inadequate towards society, exhibit relationship problems, and physically dislike themselves. Gradually, the symptoms become psychosomatic causing headaches or stomach pains, and they begin to have absences from school or university becoming progressively chronically ill ([4], p. 82).

The developing isolation from reality to escape to artificial paradises leads to increasingly artificial and selfish relationships that occur exclusively on the web or on social networks as they can exclude the need to meet a person anymore: emotional voids are filled with a message, a video call, or online chat. All this is because online communication makes it much easier not to take responsibility for one's actions as it is the artificial entity that manipulates and uses people for selfish ends. In fact, on the Internet, you can represent yourself whatever way you want, and when you are unable to manage a relationship, even a work relationship, the solution is to stop responding, silence WhatsApp chats, or simply block the user you do not know how to deal with anymore.

### 5.3. Digital Sexuality

The example of virtual isolation just discussed is daunting but, in a certain sense, not unexpected. At the same time, there is now a phenomenon that has become quite widespread and is destined for further diffusion, that of digital sexuality. Although it is an incomprehensible concept to most people, it has already climbed several steps of the Overton window. *Digisexuals* are people who choose to have sex only with a robot, without having intercourse with humans. Today, the high-tech sex industry already has a turnover of approximately 30 billion dollars a year and is a constantly growing market. “In the future, we will see the growth of human intercourse experienced entirely online. And some will begin to prefer technologically advanced virtual sex to sex with humans. We may also see more people living alone spending more time in virtual reality; a phenomenon that, as we have reported, is already happening with the Hikikomori” [6].

The first prototypes are already available on the market and interact with human beings to the point of being able to replace them not only in bed but also in more unsuspected roles. In Italy, more precisely in Turin, the first brothel where the paying customer can be with humanoid-like dolls, or rather, silicone prostitutes supplied by the Lumi Dolls ([7]), a company opened in September 2018. There are 8 dolls, which are very realistic reproductions of life-sized young women, whom you can seclude with alone or in a group (e.g., stag parties) to have sex for a fee. Reservations are made on the Lumi Dolls website and are often sold out for several months. The clients include couples and single women, and they can also choose in advance which dolls to use and which clothes they will wear.

At the moment, the site is temporarily closed for strictly administrative and fiscal reasons, as it is not exactly a shop but more like a hotel by the hour, therefore subject to different types of regulations.

This example tells us that we are on the verge of a new cultural and anthropological transformation: not only do old jobs, old roles, and old values seem destined to disappear, but man himself, or at least as we know him. Future relationships between humans and robots could have this unexpected twist that is rarely talked about, but whose impact could be very significant. In fact, as well as silicone dolls, there are also real sex robots fabricated in models for all tastes and all budgets. For example, on the market, there is Harmony, a Realbotix sex robot model, equipped with artificial intelligence, movement capacity, and its own personality [8], due to the software it is provided with that allows one to shape its personality and features, choosing from intelligent, romantic, moody, shy, and enterprising versions (he quotes). There are also male and transgender dolls as well as hybrids, i.e., with some removable parts ([8]).

Nothing can scandalize or surprise us: by now, we have learned that any idea, even the most bizarre, has an opportunity to be discussed and become reality as shown by the Overton window. Cinema floods the masses with well-calibrated messages, getting them gradually used to the scenarios that one wants to impose causing a “gentle indoctrination.”

Sadly, there is very little scientific research investigating the social, legal, and moral implications of relationships with robots In large part because they are considered vulgar and sensationalist themes by the academic world. Therefore, technology goes ahead in Japan, and practically, all of Asia and customs change while we tend to hide and pretend nothing has happened as if the problem did not exist (and in the meantime, brothels with robot dolls are opening up). But there is a lot of scientific research that needs to be done and a lot to investigate. In addition to the interaction between humans and robots, the important issue of privacy should be examined because some sex robots could be hacked for the purpose of collecting their users' data and information. It is not necessary to go much further: what has been said is more than enough to induce us to understand how pressing matters are concerning the applications of technoscience and what they impose on the societies of our time.

## 6. Considerations on Transhumanism and Posthumanism

The whole of the reflections presented in this paper can offer a suitable framework for some considerations regarding a currently discussed theme, *transhumanism*. In its various articulations, it represents a cultural movement that aims at revolutionizing, empowering, and improving the human being, physically and intellectually, through science and technology (genetics, regenerative medicine, hibernation, robotics, and the insertion of subcutaneous microchips are among the most common tools envisaged). In other words, it proposes profound changes in the concept of the human being as it was conceived until now [9]. (Bostrom reconstructed the possible remotest roots of posthumanism in 2003. The introduction of this term and its related concept can be credited to the biologist Julian Huxley.) Its leaders and followers represent heterogeneous contents and interests but with the common denominator of a mechanistic view of human existence according to which man is obliged to continue his evolution as if he were a machine or a device that must be continuously updated. Therefore, they seek to make the appropriate technology available to everyone to transform the human condition and improve their capabilities.

This attitude is in keeping with a general trend existing today to interpret the whole of the human being beyond “genetics” and “the brain.” When posthumanists present their program of *human enhancement*, many discussions concerning neurosciences reject the traditional image of the human being (from this point of view, transhumanism presents a certain ideological flavour (see González-Melado [10]). For example, the debate between Habermas and Sloterdijk is very eloquent because the latter advocates the dismissal of the characteristics that have traditionally served to describe *what is human* and proposes to replace them by a new conception that locates humans closer to animals from below and to machines from above (for this famous debate, let us see, for example, [11, 12]).

Transhumanists maintain that we can legitimately reform ourselves and our nature in accordance with human values and personal aspirations see, for example, (Pearce 2015) [13]. Their basic philosophical claim is the *liberation of man from biology*: this inevitably pushes us to ask what it means to be “human,” what is nature, and what is culture.

Briefly, transhumanism rejects the view of nature as something stable and unalterable and maintains that the moral value of the human being does not reside in belonging to a certain *species* but in what he *does*. Therefore, technological advances must be used for the moral improvement of humans. Posthumanists declare that this improvement will not produce negative effects since it also involves improving the *moral behaviour* of people; hence, it is not possible to think that a moral evil will be produced.

Another problem is the disparity between the *ideal image* of what we think we are (and that the posthumanists already sell us) and what we *really are*. In Western society today, many of us have problems identifying who we *truly are*, accepting our limitations, and relating them in a mature and balanced way with what we *would like to be*, i.e., with images of a particular *ideal self* determined by cultural patterns. Accepting the image that the mirror shows us when we don't like it is complicated, and a good makeover is a fantastic solution to get closer to what we would really like. Becoming a world champion in a sport is a dream that becomes more achievable if you improve your performance with the help of some type of substance. Being a music star if you don't have a beautiful voice is possible with the use of a good synthesizer. But is it our *true face* that we see with super makeup, is it *really the best* athlete that is on enhancing drugs, is it *real* that you have a beautiful voice when it has been synthesized by a device? Today, most of us will probably still answer negatively to all these questions so we conclude by a straightforward analogy: it is not true that we are going to become super men or super women when we do a lot of things, thanks to artificial devices that we incorporate into our brain or other parts of the body. We will not be super men or super women, but we will be people just as limited as we are now only we will be superbly assisted by prosthetics and artificial tools. Moreover, perhaps, we are even more limited because it is undeniable that what we do not exercise atrophies or does not even develop; thus, we lose skills and abilities that we would otherwise have at full capacity.

At this point, doubts are more than legitimate. For example, if we consider the 20th century that has just ended, in a sense, it seems the century which produced the greatest progress in the history of humanity, precisely from the outlook of progress in the various sciences (not only physical). Yet, it is also the century that has seen unprecedented forms of barbarism, including the extermination of entire populations coldly programmed and justified by aberrant ideologies, such as Nazism and Communism. We have seen wars in which opponents not only fought on battlefields but also dropped destructive bombs on the enemy's civilian population, razing cities, and even annihilating hundreds of thousands of defenceless civilians in seconds and also leaving negative consequences for their future descendants. Faced with these atrocities (as well as other critical aspects of today's technologized societies), Sloterdijk argued that the idea of the advancement of man by cultivating his spirit, his reason, and his feelings, as the philosophers of the Enlightenment had believed, has revealed to be a failure. To this idea, according to which “good reading” is what improves man, he proposed to replace the idea that a new humanism should be based on science and technology. He maintained, however, that man continues to be the owner of technoscience and knows how to use it wisely (or with *prudence* in the Aristotelian sense). But it is difficult to carry out this project by relying on science and technology alone as they completely ignore the difference between *being* and *ought to be.* For this reason, as we have pointed out, Sloterdijk finally proposed an image of man intermediate between animals and machines, in which what is specifically human is lost. Therefore, when the application of technology to the modification of human nature itself begins to be considered, all perplexities resurface since at this point man would no longer be the wise user of technoscience, but the very random and unpredictable result of the blind growth of the latter [12] (Elena Postigo has given a significant portrayal of the posthumanist conception: “from the bioethical point of view, the most serious implications of the realization of this theory are: the eugenic elimination of “imperfect” human beings or those with malformations (eugenic abortion and pre-implantation diagnosis for selective purposes), the creation of “more perfect” human embryos, the elimination of equality between all human beings, the use of nanotechnology with human applications without thinking beforehand about its consequences for man (think, for example, of deprivation, impediment or control of freedomand conscience), the cryopreservation of the human being, etc. In addition, basically, the increase of a reductionist mentality regarding man, efficient and not respectful of the dignity of the human being in any situation that he may encounter” ([14], p. 281). In such way, the original meaning of “posthumanism” that simply amounted to abandoning the ideals of the classical “humanities” evolved into the idea of a “transhumanism”, i.e., of a “transition” towards an undetermined end, which in any case was condemned to be a posthumanist unpredictable horizon in which the *human* would be hardly recognizable. No one doubts the goodness of scientific progress in the fields of health, education, and such like, but here, the intention is to *change the human species*, and by beyond humanism, some scholars already think of posthumanism in the second sense outlined above: a stage where humanism has been left behind.

## 7. Conclusion

The critical considerations about posthumanism and transhumanism have highlighted the limits of those conceptions in which the value of man and his existence is measured exclusively on the basis of what science and technology can offer. The inadequacy of these resources does not only consist in the fact that they point to an uncertain future that we have just described as negative consequences of the most recent advances in information technologies. In the case of digital sex, which could be considered an amazing achievement, the sterility of reducing sexuality to pure physical pleasure emerges, not only by ignoring its connection to the sphere of love and what that means to man but even lowering it below what it implies at the basic level of the animal world. This is why the due appreciation of science cannot be separated from an appropriate investigation of values.

Among the various types of values, those of a moral nature are particularly significant for the purposes of this paper. Each technological advancement addresses only one particular problem but does not help to solve the others related to it. The situation of the current pandemic mentioned at the beginning of this paper clearly attests to this. In the early days, when doctors were trying to learn about the strain of the virus in order to fight it, the only remedy that could be used was to limit the spread of the contagion through strict lockdown measures that forced millions of people to remain isolated at home for entire weeks, and this implied the sudden interruption of many productive activities with great economic damages and loss of jobs. Many were under the illusion that science would solve the problem by producing a vaccine. However, even after this “miracle” was obtained many months later, it was evident that not only the implementation of this tool would still take a long time, but that the gravity of the situation had degenerated. Core factors causing this decline are linked to inadequate health structures, even in the most advanced countries, and to different social, economic, and cultural conditions that no vaccine can affect.

For example, for many families, the loss of work has meant the risk of dying of hunger, which is almost equivalent to the risk of dying from contagion, and has often led to acts of violence, whereas the rediscovery of the ethical value of *solidarity* contributes to making people more effective in the fight against the pandemic. This forces us to reflect on the many aspects of human *vulnerability* that are not reduced to mere physical health and which we too easily choose not to acknowledge. Working for a better future for man is a great stimulus to our moral conscience yet not by trying to “enhance” his nature with technological interventions or even genetic manipulations but by discovering the richness and roots of his dignity in his interiority as an individual person and as a member of the great human brotherhood of man.

## Data Availability

No data were used to support this study.
